The article "Astrocytes Protect Human Brain Microvascular Endothelial Cells from Hypoxia Injury by Regulating VEGF Expression" was published in 2022. Journal: J Healthc Eng.

# Astrocytes Protect Human Brain Microvascular Endothelial Cells from Hypoxia Injury by Regulating VEGF Expression

**DOI:** 10.1155/2022/1884959

**Published:** 2022-03-18

**Authors:** Jianmin Liu, Jiwen Li

**Affiliations:** ^1^Department of Neurosurgery, Affiliated Hospital of Shandong University of Traditional Chinese Medicine, Jinan, Shandong 250011, China; ^2^Department of Neurosurgery, Zhangqiu District People's Hospital, Jinan, Shandong 250200, China

## Abstract

Hypoxic-ischemic stroke has been associated with changes in neurovascular behavior, mediated, in part, by induction of the vascular endothelial growth factor (VEGF). The objective of this study was to investigate the effects of human astrocytes on the proliferation, apoptosis, and function of human microvascular endothelial cells (hBMEC) in vitro. Human microvascular endothelial cells (hBMEC) and human normal astrocytes (HA-1800) were used to establish in vitro cocultured cell models. The coculture model was used to simulate hypoxic-ischemic stroke, and it was found that astrocytes could promote hBMEC proliferation, inhibit apoptosis, reduce cell damage, and enhance antioxidant capacity by activating the VEGF signaling pathway. When VEGF is knocked out in astrocytes, the protective effect of astrocytes on hBMEC was partially lost. In conclusion, our study confirms the protective effect of hBMEC and laid a foundation for the study of hypoxic-ischemic stroke.

## 1. Introduction

Hypoxic-ischemic stroke refers to cerebral ischemia and hypoxia injury caused by vascular obstruction, which leads to focal or whole-brain dysfunction. It is characterized by high morbidity, high disability rate, high mortality rate, and high recurrence rate and seriously endangers human health [1]. Hypoxic-ischemic stroke occurs in the absence of blood flow of oxygen and nutrients [2]. As the body will undergo angiogenesis to restore blood flow when it lacks blood flow, angiogenesis is essential for the repair of hypoxic-ischemic stroke. Despite significant improvements in medicine and intravascular recanalization, treatment options for hypoxic-ischemic stroke remain limited [3, 4]. Therefore, the promotion of angiogenesis is considered to be an effective therapeutic target for hypoxic-ischemic stroke [5]. A deeper understanding of the of angiogenesis after hypoxic-ischemic stroke will help to facilitate the arrival of such therapies.

Coculture is to mix and coculture two kinds of cells, so that the morphology and function of one kind of cells can be expressed stably and maintained for a long time. It has been found that the cotransplantation of neural stem cells and olfactory nerve sheath cells can attenuate the apoptosis of rat neurons, promote the survival of host neurons, and promote neuronal recovery in traumatic brain injury through anti-inflammatory mechanisms [6]. The coculture and transplantation of umbilical cord blood pluripotent stem cells and lymphocytes can improve the symptoms of neurological defects, reduce the volume of cerebral infarction, and alleviate the inflammatory response of ischemic brain death rats [7]. Coculture of endothelial progenitor cells and neural progenitor cells increased VEGF expression and activated the PI3K/Akt pathway, synergically protecting brain endothelial cells from hypoxia/reoxygenation-induced injury [8]. The BMECs and astrocyte coculture model is the most widely used the in vitro BBB model. Astrocytes have been found to support neuronal repair and participate in and maintain the blood-brain barrier properties of BMECs. Coculture of hCMEC/D3 with astrocytes reduces paracellular permeability to enhance the ability of the blood-brain barrier to screen for neurotoxicity [9]. However, the effect of astrocytes on the proliferation and apoptosis of hBMEC and its mechanism remain unclear.

Angiogenesis refers to the formation of new blood vessels from the differentiation of vascular endothelial cells of existing capillaries and posterior capillary venules [10]. Angiogenesis after brain injury can promote the recovery of neurons and brain functions, so the study of angiogenesis is of great significance in brain injury. During this process, astrocytes are involved in the regulation of endothelial cell growth, the regulation of tight junctions between endothelial cells and the chemotaxis of phagocytes [11]. After brain injury, astrocytes play a double-edged role. On the one hand, excessive activation produces a large number of inflammatory mediators leading to cell injury. On the other hand, various neurotrophic factors are secreted to activate the proliferation of endogenous neural stem cells and directly affect the repair of injured cells and nerve regeneration [12, 13]. In addition, astrocytes themselves also secrete factors that promote nerve production in vitro, such as the epidermal growth factor, basic fibroblast factor, brain-derived nerve growth factor, insulin-like growth factor, and vascular endothelial growth factor [14, 15]. It has been found that under hypoxic conditions, induction of VEGF mRNA and protein in cerebral astroglial cultures occurs [16, 17]. However, the mechanism of interaction between cerebral microvascular endothelial cells and astrocytes under hypoxia remains unclear.

In this study, we established an in vitro coculture model of human astrocytes and human brain microvascular endothelial cells by the transwell technique to observe the effects of astrocytes on proliferation, apoptosis, and antioxidant capacity of hypoxia-mediated brain microvascular endothelial cells. These results lay a foundation for further study on the protective mechanism of astrocytes against brain microvascular endothelial cells and provide a potential treatment for hypoxic-ischemic stroke.

## 2. Materials and Methods

### 2.1. Cell Culture

hBMEC and HA-1800 cells (FuHeng Cell Bank, China, Shanghai) were cultured in the DMEM medium containing 10% FBS and 1% double antibody, and the medium was changed every 2 days. Normally, cells were maintained in an incubator filled with 95% air and 5% CO_2_ at 37°C. For hypoxia treatment, hBMEC was incubated in a hypoxic incubator filled with 94% N_2_, 5% CO_2_, and 1% O_2_ at 37°C.

### 2.2. Coculture of hBMEC and HA-1800

hBMEC was digested by trypsin to prepare a single cell suspension with a cell density of 2 × 10^5^/L and inoculated on a 24-well plate. A noncontact cell coculture system was established using transwell cells. HA-1800 trypsin was digested into a single cell suspension with a cell density of 2 × 10^5^/L. The suspension was inoculated on the underside of the transwell cells coated with collagen type I, and then, the cells were placed in the pores inoculated with hBMEC. For hBMEC cultured separately, no compartment was inserted into the hole.

### 2.3. Cell Viability by CCK-8

Cell viability was determined by CCK-8 assay (Sigma-Aldrich, St. Louis, MO, USA). In short, cells were digested and removed from each group, and hBMEC were planted in 96-well plates and incubated for 2 hours at 37°C in 100 ul DMEM containing 10 ul CCK-8 solution. Absorbance at 570 nm was measured on a microplate reader (Bio-Rad, Hercules, CA, USA). All experiments were performed three times.

### 2.4. TUNEL

The coculture model of hBMEC and HA-1800 was established by the Transwell technique. In normoxic (5% CO_2_, 95% air) and hypoxic (1% O_2_, 5% CO_2_, 94% N_2_) conditions, the cells in the culture group and the VEGF knockout group were fixed after specified treatment. Then, fixed and permeabilized with 4% paraformaldehyde and 0.1% triton X-100, hBMEC were incubated with the TUNEL reaction mixture for 1 hour at 37°C in the dark and stained with DAPI for 15 minutes. Confocal laser scanning microscopy (FV300, Olympus, Japan) was used to detect the fluorescence of the cells.

### 2.5. Knockdown of VEGF with siRNA

The siRNA specifically targeting VEGF was designed and constructed by Geneseed (Guangzhou, China). The sequences of siRNAs used were as follows:

HA-1800 was transfected with certain vectors using Lipofectamine 2000 (Invitrogen) in accordance with the manufacturer's instructions and then was used for further experiments. Western blot analysis confirmed the specific silencing of VEGF expression.

### 2.6. Superoxide Dismutase (SOD) Assay

The cells treated by different groups were digested, and the cell suspension was lysed with RIPA ice for 15 min, 12000 rpm at 4°C, and centrifuged for 10 min. The supernatant was collected, and the content was determined using the SOD kit (Nanjing Jiancheng Bioengineering Institute).

### 2.7. Western Blot

After the indicated treatment, hBMEC were collected and lysed in RIPA lysis and extraction buffer (Thermo Fisher Scientific, Waltham, MA, USA). Protein concentrations were evaluated by the BCA method (Micro BCA Protein Assay Kit, Thermo Fisher Scientific), and 50 *μ*g of each sample was separated by SDS-PAGE on a 12% gel. Then, the proteins were transferred to PVDF membranes (Millipore, MA, USA). After blocking with nonfat milk, the membranes were incubated with a primary antibody overnight at 4°C, washed, and then incubated with a secondary antibody for 1 h each at room temperature. The antibodies used were anti-VEGF (ab32152), ERK (ab17942), p-ERK (ab50011), Akt (ab8805), p-Akt (ab38449), and goat anti-rabbit secondary antibody (ab150077). The results were quantified, and the images were processed using ImageJ software. GAPDH was used as an internal loading control.

### 2.8. Statistical Analysis

Statistical analysis was conducted using SPSS 16.0 software (SPSS Inc., Chicago, IL, USA). The measurement data are expressed as mean ± SD and were subjected to statistical analysis using one-way analysis of variance (ANOVA). When significant interactions were detected in any ANOVA paradigm, *t*-tests were used to demonstrate effects between individual groups. Values of *P* < 0.05 were considered statistically significant.

## 3. Result

### 3.1. Establishment of the Coculture Model of Astrocytes (HA-1800) and Human Microvascular Endothelial Cells (hBMEC)

In order to investigate the effect of astrocytes on hBMEC, transwell technology was used to establish the indirect coculture model of HA-1800 and hBMEC in vitro. Cells inoculated with HA-1800 were removed at 0 h, 6 h, 12 h, and 24 h under normoxia to detect the effect of coculture of astrocytes at different times on hBMEC. First, CCK-8 assay showed that HA-1800 significantly increased hBMEC proliferation activity over time (Figure 1(a)). Next, superoxide dismutase (SOD) level, an antioxidant index, was detected in cell lysates, and the results showed that the SOD level increased over time (Figure 1(b)). At same time, TUNEL observed that the addition of HA-1800 significantly inhibited apoptosis (Figures 1(c) and 1(d)).

### 3.2. Coculture of HA-1800 and hBMEC Promoted Functional Repair of Brain Microvascular Endothelial Cells under Hypoxia

The structure and cell base of blood-brain barrier (BBB) are brain microvascular endothelial cells (BMEC). The tight connection between endothelial cells is the fundamental guarantee of BBB's characteristic structure and maintenance of barrier function. Endothelial cells are often the direct target cells of pathological damage factors such as hypoxia, and hypoxia will bring a series of changes in the internal environment of cell growth [18–21]. To investigate the effect of astrocytes on hBMEC under hypoxic conditions, we cocultured HA-1800 and hBMEC under normoxic and hypoxic conditions for 24 h. It was found that the proliferative activity and SOD levels of hBMEC cells were significantly lower under hypoxia compared to normoxia. However, coculture with astrocytes under both normoxia and hypoxia significantly enhanced the proliferative activity and SOD levels of hBMEC (Figures 1(a) and 1(b)). Next, TUNEL observed that hypoxia promoted hBMEC cell apoptosis, while coculture reversed hypoxia-induced apoptosis (Figures 2(c) and 2(d)). In conclusion, we found that HA-1800 can significantly enhance hBMEC cell activity under normoxia, and coculture of HA-1800 and hBMEC can repair cell function damage caused by hypoxia.

### 3.3. HA-1800 Affects hBMEC Function through VEGF Signaling Pathway

VEGF signaling pathway plays an important role in the process of angiogenesis [22]. We speculated that coculture may promote hypoxia-induced angiogenesis through the VEGF pathway. In addition, ERK and Akt pathways are key intracellular signal transduction pathways for angiogenesis after activation of the VEGF signaling pathway [23]. Therefore, we also studied the effects of coculture on the regulation of ERK and Akt pathways under hypoxia. Western blot was used to detect the protein levels of related pathways, and it was found that the expression of VEGF and the phosphorylation of ERK1/2 and Akt increased in both the coculture group and hypoxia treatment for 24 h. This induction was more significant in the hypoxia coculture group than in hypoxia or coculture only (Figures 3(a) and 3(d)). Overall, our data indicate that VEGF signaling pathway can be activated in both coculture and hypoxia, with the induction of HA-1800 and hBMEC being more significant in hypoxia.

### 3.4. Knockout of VEGF in HA-1800 Can Eliminate the Effect of Hypoxia on the Functional Integrity of hBMEC Cells

To establish a causal relationship between the production of cell-derived VEGF in HA-1800 and hypoxia-induced hBMEC dysfunction, we used siRNA methods to knockout VEGF in HA-1800. Western blot analysis confirmed specific silencing, showing a more than 80% reduction in the level of HA-1800 VEGF protein transfected with VEGF siRNA (Figure 4(a)). Most importantly, VEGF knockout significantly reduced cocultured-induced cell proliferation, inhibition of apoptosis, and antioxidant capacity under hypoxia (Figures 4(b)–4(d)). These results suggest that HA-1800 may protect the functional integrity of hBMEC through VEGF in hypoxia.

## 4. Discussion

Acute blood-brain barrier (BBB) disruption occurs in the first few hours of hypoxic-ischemic stroke and has received increasing attention. BBB is composed of endothelial cells arranged on the cerebral microvessels, and the peripheral cells, basal membrane, and foot processes of astrocytes outside the endothelial cells also participate in BBB formation [24, 25]. It has certain barrier structures that limit the ability of substances to pass through, regulate, and maintain the stability of the central nervous system microenvironment [26]. At present, it is the most common method to construct the blood-brain barrier model of ischemic stroke by coculture of animal primary endothelial cells and glial cells [27]. It has been found that the expression level of *γ*-GT enzyme decreased significantly during the passage of primary cells, suggesting that cells may gradually lose some BBB characteristics during primary culture [28]. The use of passage cell lines is cost-effective, fast, and allows for extensive experiments by passage and proliferation of cells without the need for responsible cell separation. Therefore, in this study, representative human cerebrovascular endothelial cell line hBMEC and human positive astrocyte HA-1800 were cocultured to establish in vitro BBB, and the effect of hypoxia on BBB was evaluated.

After brain injury, the blood-brain barrier is hypoxic and ischemic. In this state, brain microvascular endothelial cells are affected by astrocytes and various angiogenesis factors during hypoxia. At the same time, angiogenesis-related growth factors and cytokines secreted by glial cells are regulated by hypoxia-inducible factors, and activation of hypoxia-inducible factors induces the tolerance of glial cells to ischemic hypoxia [29]. Vascular endothelial growth factor (VEGF) is one of the most important proangiogenic factors in the microenvironment of choroidal angiogenesis. A large number of studies have confirmed that VEGF plays a key role in the process of pathological neovascularization [30]. As a specific mitogen of endothelial cells, VEGF can induce the division and proliferation of vascular endothelial cells and promote the migration of endothelial cells, which is conducive to the formation of a large number of blood vessels by budding of new vessels. Brain microvascular endothelial cells, pericytes, and astrocytes can produce VEGF. In the state of hypoxia, analyzing the intracellular environment of cerebral microvascular angiogenesis from the cellular level, it can be found that vascular endothelial cells are regulated by a variety of surrounding cells [31], one of which is AS cells. The hypoxia-regulated nature of VEGF makes it an important neovascularization factor, which can specifically bind to vascular endothelial cells and promote the growth of endothelial cells, thus participating in hypoxia-induced choroidal neovascularization. It has been found that both hypoxia and astrocytes can promote VEGF expression [16, 17]. We detected the protein expression level of VEGF by Western blot and obtained consistent results. The expression of VEGF in hBMEC increased under hypoxia or coculture, and the increase of VEGF expression was more significant when hypoxia and HA-1800 were cocultured at the same time. Meanwhile, when VEGF is knocked out in HA-1800, ha-1800 loses part of its protective function against hypoxia injury. These results suggest that HA-1800 may affect the proliferation, apoptosis, and antioxidant capacity of hBMEC by regulating the expression of VEGF.

In conclusion, our results confirm the important role of astrocytes in mediating ischemia barrier damage. We found that under normal conditions, coculture of HA-1800 and hBMEC significantly increased cell proliferation activity, inhibited apoptosis, and promoted ROS. Under hypoxia, the proliferation activity of hBMEC cells decreased, apoptosis cells increased, and intracellular ROS level decreased, while coculture could partially reverse the cell damage caused by hypoxia. This function may be related to ERK and Akt phosphorylation and VEGF protein expression. We knocked out VEGF in astrocytes and significantly reduced their ability to resist hypoxia injury. These results suggest that astrocytes can protect hBMEC from hypoxia injury by activating the VEGF signaling pathway.

## Figures and Tables

**Figure 1:** Effect of HA-1800 on hBMEC in coculture at various times. (a) The effect of coculture on hBMEC cell proliferation at various times detected by CCK-8. (b) The change of SOD in homogenate of cocultured hBMEC cells at various time detected by the kit. (c)-(d) The effect of coculture at various times on hBMEC cell apoptosis detected by TUNEL.

**Figure 2:** HA-1800 protects hBMEC cells from hypoxia damage. (a) The effect of coculture of HA-1800 on the proliferation activity of hBMEC under 24 h hypoxia treatment detected by CCK-8. (b) SOD content in lysate of hBMEC cells detected. (c)-(d) The effect of HA-1800 coculture on hBMEC apoptosis under hypoxia treatment for 24 h detected by TUNEL.

**Figure 3:** Effect of coculture on VEGF signaling pathway-related proteins. (a)–(d) The effect of coculture of HA-1800 and hBMEC on VEGF protein level detected by Western blotting and statistical analysis of Western blotting. Phosphorylation levels of the indicated kinases ERK1/2 and Akt were also quantified by densitometry.

**Figure 4:** HA-1800 protects hBMEC by VEGF. (a)-(b) Western blot to detect the transfection efficiency of knockout VEGF in HA-1800 cells. (c) The effect of VEGF knockout in HA-1800 cells on hBMEC proliferation activity under hypoxia detected by CCK-8. (d) To detect the effect of VEGF knockout on hBMEC apoptosis in HA-1800 cells under hypoxia through TUNEL. (e)-(f) To detect the effect of VEGF knockout in HA-1800 cells on SOD in hBMEC cell lysates under hypoxia.

## Data Availability

The data used to support the findings of this study are available from the corresponding author upon request.
